The article "Realization of Super-Large-Diameter Slurry Shield Passing through Settlement-Sensitive Area Based on Unreinforced Disturbance Control Technology" was retracted in 2023. Reasons: unreliable results or conclusions; concerns about the data; concerns about the peer review; concerns about the citations.

# Realization of Super-Large-Diameter Slurry Shield Passing through Settlement-Sensitive Area Based on Unreinforced Disturbance Control Technology

**DOI:** 10.1155/2022/6299645

**Published:** 2022-01-13

**Authors:** Dongshuang Liu, Xinrong Liu, Zuliang Zhong, Yafeng Han, Fei Xiong, Xiaohan Zhou

**Affiliations:** ^1^School of Civil Engineering, Chongqing University, Chongqing 400045, China; ^2^National Joint Engineering Research Center of Geohazards Prevention in the Reservoir Areas (Chongqing) of Chongqing University, Chongqing 400045, China; ^3^Key Laboratory of New Technology for Construction of Cities in Mountain Rrer of Chongqing University, Chongqing 400045, China

## Abstract

Due to the complex construction conditions of shield tunnels, ground disturbance is inevitable during the construction process, which leads to surface settlement and, in serious cases, damage to surrounding buildings (structures). Therefore, it is especially important to effectively control the constructive settlement of subway tunnels when crossing settlement-sensitive areas such as high-density shantytowns. Based on the project of Wuhan Metro Line 8 Phase I, the shield of Huangpu Road Station-Xujiapang Road Station interval crossing high-density shantytowns, we study the disturbance control technology of oversized diameter mud and water shield crossing unreinforced settlement-sensitive areas during the construction process. By optimizing the excavation parameters and evaluating the ground buildings, the excavation process can be monitored at the same time, and the water pressure, speed, and tool torque required during the excavation during the construction process can be finely adjusted; the control of tunneling process parameters can provide reference and basis for analyzing the construction control of large-diameter shield through old shantytowns.

## 1. Introduction

With the rapid development of urban rail transit construction, complex situations such as mud-water balanced shield crossing complex strata and dense old building complexes are becoming more and more frequent [1–3]. Around the settlement control of tunnel shield under old buildings, many useful studies have been done by domestic and foreign research scholars in different engineering contexts [4]. After a long investigation on the stability and settlement law of the upper buildings during the shield underpass, it is concluded that in general, the surface settlement of the upper buildings accounts for 30% to 90% of the total amount during the shield underpass. Wang et al. [5] studied the influence of the tunnel shield excavation process on the settlement of the upper structures under different burial conditions. Charaniya, Nassar, and Al-Mahdi [6, 7] studied the problem of surface settlement and deformation; that is, when the actual site water pressure is high, the water storage tunnel encounters soil particles with strong water permeability. Rho et al. and Reed et al. [8, 9] simplified the calculation method for such problems and simplified the complex three-dimensional problem into a planar problem, which greatly reduced the calculation volume and accelerated the calculation process.

People's living space is getting more and more crowded, and traffic congestion is becoming more and more prominent. The rational exploitation of underground space can greatly help to relieve the pressure of urban traffic, and the development of underground rail transportation has become one of the important directions for sustainable social development [4, 10]. China is developing rapidly in urban rail transit construction and currently ranks first in the world in total subway construction.

In urban metro construction, tunnel construction mainly includes the open cut method, shield method, and mining method. Due to the advantages of short construction time, high engineering safety, high automation, and low impact on the surrounding environment [11], shield method construction has now gradually replaced other methods as the first choice for urban metro construction. The shield method construction process is a process in which the shield machine excavates and digs forward in the underground soil layer, and the shield shell and tube sheet are used to maintain the stability of the soil around the excavation and avoid excessive soil deformation, while the soil is excavated by the cutting device in front of the excavation, and the cut down soil is cut by the shield machine [12]. The excavation is carried out by the cutting device in front of the excavation, and the cut soil is transported out of the hole by the excavation machine inside the shield machine. The jack at the end of the shield acts on the completed tube sheet, and the jack pushes the shield forward while the tube sheet is released from the end of the shield to form the tunnel structure. During the tunneling process, as the diameter of the cutter plate and the outer diameter of the shield excavated in front of the shield are larger than the outer diameter of the tunneled pipe pieces inside the shield, when the pipe pieces are assembled and completely disengaged from the tail of the shield machine, an annular gap will be formed between the pipe pieces and the soil layer, which is called the shield tail gap [13].

Usually, post-wall grouting is used to fill the void at the end of the shield, and the post-wall grouting construction technology is simple and has good engineering effect. Therefore, it is widely used in tunneling and other geotechnical engineering. Post-wall grouting is relatively mature; however, the movement of the slurry in the shield tail void is complicated. There is still a lot of disagreement in the form of pressure distribution for post-wall grouting in shield tunnels. There are still many differences in the form of pressure distribution, and the mechanism of slurry action with the surrounding strata and tube sheet is still to be investigated. Therefore, the mechanism of post-wall grouting has been a topic of interest for many researchers and scholars [8, 14]. The current grouting studies are basically for small and medium-sized shield structures, and the effect of gravity on the grouting pressure is not considered, but the effect of gravity on the grouting pressure of large-diameter shield structures cannot be ignored. Therefore, it is necessary to analyze the construction process of post-wall grouting of large-diameter mud and water shield [15].

This study takes the Wuhan Rail Transit Line 8 Huangpu Road Station-Xujiapang Road Station river-crossing shield tunnel project as an example and proposes construction control techniques for shielding crossing-sensitive areas in dense shantytowns based on a brief analysis of the project background and key difficulties.

## 2. Related Work

The history of behind-the-wall grouting was developed as part of geotechnical grouting for shield tunneling applications, which opened the door to the use of grouting in geotechnical engineering in 1802 when Charles Berigny, a French civil engineer, used manual hammering to inject clay and lime into the ground by means of a wooden impact cylinder device when dealing with sand gates. Zaslow et al. [16] from the Research Institute of China Railway Tunneling Group developed a new type of single-liquid slurry, which has a long setting time of more than 3–12 h and can be adjusted to adapt to different geological conditions and construction situations. By selecting different water-reducing agents for the test, Qiang et al. [17] improved the pumpability of the slurry, improved the stability of the slurry, improved the construction performance of the post-wall synchronous injection slurry, and obtained a good grouting effect.

In the tunneling project of Beijing Metro Line 5, Zhou et al. [18] studied the composition of the slurry, and finally the inert slurry was selected for the slurry used in the construction, which is based on quicklime and fly ash as the main ingredients, and a patent was published for this slurry. The slurry has the characteristics of low manufacturing cost, simple ingredients, good compatibility, and easy production and also has the advantages of preventing leakage from the longitudinal joints of the pipe sheet ring, convenient construction management, and less ground settlement. Liu et al. [19] conducted a lot of research on the admixtures of post-wall grouting materials. Usually, synchronous grouting materials contain bentonite compounded with water-reducing agent, and Li et al. [20] found that the grouting effect is better with the choice of water-retaining agent compared to water-reducing agent, and the cost of both is similar, so the water retaining agent is worth using widely. For post-wall slurry material delivery, Lai et al. [21] invented modified lignin efficient grouting pumping agent which can improve the stability and water-reducing enhancement of slurry while reducing the pumping resistance of slurry and improving its strength, so that the slurry has a proper setting time.

In the South-North Water Transfer Central Line crossing Yellow River Tunnel Project, Xie et al. [22] studied how to optimize the ratio of grouting materials based on the experimental principle of uniform design for fine sandy soils and compared and analyzed the slurry performance influenced by each component of the single-liquid active grouting material.

For the effect of post-wall grouting, the first research in this area was carried out and some results were obtained by the whole group led by Professor Huang Hongwei from Tongji University. In a subway shield tunnel project in Shanghai, Qiu et al. [23] studied the deformation properties and longitudinal mechanics of shield tunnels, paying special attention to the effect of behind-wall synchronous grouting, and for the first time used ground-penetrating radar method to detect the distribution of tunnel synchronous grouting slurry, proposing that the form of behind-wall slurry distribution of the tube piece can be effectively detected by this method, which provides the control of longitudinal mechanical deformation properties of tunnel grouting, laying the foundation for the longitudinal mechanical deformation control of tunnel grouting.

Field measurements of the tube lining pressure revealed that the dissipation time of the grouting pressure has a significant effect on the variation of the tube lining pressure. For 9.5 m diameter shield tunnels, Huang et al. [24] conducted a field experimental study on simultaneous post-wall grouting. After analyzing the field monitoring data, it was found that the surface settlement was significantly affected by the grouting pressure, and the distribution of the grouting pressure in the cohesive soil was found to be small at the top and large at the bottom when the shield was stopped. In order to achieve accurate measurement of the pressure effect of post-wall grouting on the pipe sheet lining, Yin et al. [25] developed a gasket type lining pressure measurement meter, which is capable of long-term uninterrupted monitoring of the pipe sheet pressure as well as the pressure of the grouting layer. Analysis of the field monitoring data revealed that the main reason for the change in pipe sheet pressure was the change in grouting pressure. Meschke [26] took the surrounding rock of a project shield tunnel as the object of study and used field monitoring method for this surrounding rock pressure, illustrating the selection and burial of measuring elements required for monitoring, testing methods, and analysis of test results. Li and Yuan [27] used monitoring instruments to measure the dry shrinkage stresses applied to the tube sheet lining, the post-wall grouting tube sheet lining stresses, the tube sheet lining stresses after stabilization of the grouting ring, and the surrounding rock pressure in the shield tunnel during construction. The corresponding analytical solutions were obtained by using the steel stress back calculation formula combined with the monitoring data for the annular pressure of the pipe sheet and the bending moment. In [28], the interaction between the tube sheet and the surrounding soil in a shield tunnel through old loess was studied by means of real-time on-site tracking and monitoring.

Through a model test study of post-wall grouting, Zhao et al. [29] found that tunnel pressure loads and soil displacements were significantly influenced by grouting pressure and soil density. In the centrifugal model test, Meng et al. [30] used a mini-shield machine to simulate the shield boring process, including the release of the tube sheet lining from the shield tail, for shield tunnels with different burial depths with or without shield tail voids and derived the deformation of the surrounding strata and the variation of the soil pressure on the top of the tube sheet. Zhang et al. [31] conducted an experimental study using a homemade behind-the-wall grouting test device to study the deformation of the grouted body and the variation of the grouting pressure considering the grouting material, the grouting pressure, and the geological conditions and concluded that the surface settlement was significantly affected by the grouting pressure and the geological conditions. Many physical model tests of post-wall grouting were conducted by Merceron and Prouteau [3], and it was found that the soil pressure distribution was significantly influenced by the grouting pressure and soil compaction. The shield tunneling in loose sand and dense sand layers was studied separately.

In [4], the slurry diffusion radius and the pressure applied to the pipe sheet were calculated for the slurry under two conditions, considering viscosity and not considering viscosity, respectively. Wang et al. [5] established a three-dimensional finite element model for mud-water balanced shield tunneling, in which the soil was simulated by elastomer, the lining was simulated by shell unit, and the slurry injection was simulated by solid unit, and the support pressure was applied at the excavation surface during shield tunneling, and the slurry injection pressure was considered at the shield tail gap, and the effects of the support pressure and slurry injection pressure on the ground displacement were analyzed.

## 3. Project Overview

Located 450 m upstream of Wuhan Yangtze River Second Bridge, the Wuhan Rail Transit Line No. 8 Phase I civil construction tunnel project, Huangpu Road Station-Xujiapang Road Station, is a 12.1 m diameter single tube double line composite lining shield tunnel. The shield interval is 3.185.5 m long. After the longitudinal section of the river-crossing line leaves Huangpu Road Station, the line descends with a longitudinal slope of −18.4‰ and a slope length of 1,710 m. It reaches the lowest point of the river line with a gentle slope of +4.8‰ and a slope length of 420 m. It then ascends with a slope of +27.49‰ and a slope length of 952.708 m to Xujiapang Road Station [14].

The shield traverses the stratum as shown in Figure 1. The shield traverses 1.820 m of full-section fine sand strata and 1.365 m of soft and hard composite strata with a maximum compressive strength of 24.5 MPa of cemented rocks.

The shield tunnel starts from Xujiapang Road Station with a radius curve of *R* = 700 m and crosses a high-density shantytown (DK12 + 185.000-DK12 + 939.618, total length of 754.618 m) for a long distance, mainly passing through buildings (structures) such as Wumen Village, Station New Village, Xujiapang Street, Chengsanli, and other villages with 1 to 4 floors, with a total of 140 houses passing underneath and 308 houses passing sideways, part of which is shown in Figure 2. Most of these houses were built before the 1990s, and the appearance of these buildings is old and obsolete, and most of them have to peel walls and cracked walls, which are serious safety hazards. Figure 2 shows the plan of Huangpu Road Station-Xujiapang Road Station through some shantytowns.

## 4. Construction Control Key Technology

### 4.1. Pre-Digging Settlement Control Technology

Before the assessment of existing buildings and safety standards were formulated. Relevant units were commissioned to conduct a safety risk assessment of existing buildings along the shantytown. This interval has 2 level-1 environmental risk projects, and the main measures for shield construction through the level-1 risk project profile are as follows: 15 m range on each side of the tunnel centerline over the risk source is the strongly affected area, and the residents in the houses in the area are to be transitioned before the construction of the interval; the interval across the river crosses the railroad track and cross-line flyover at Wuchang North Station in Wuchang section, and pre-reinforcement measures (cuff tube grouting, rotary piles, and three-row composite anchor piles) are taken before the construction for the construction of the interval.

The initial 75 m of shield advance was used as the test section, and the shield boring parameters were continuously adjusted during the shield boring process based on real-time monitoring. The construction parameters of the shield in the section under the old shantytown are shown in Table 1.

During the shield tunneling process, the shield machine controls the tunneling attitude and adjusts each tunneling parameter in real time according to the generated ground settlement to ensure the safety and stability of the surrounding soil during the construction process, for example, the relationship between the pressure difference between the inside and outside of the soil layer and the ground settlement is shown in Figure 3.

## 5. Analysis of Digging Parameters

The geological condition and surrounding environment are important parameters in the process of shield tunneling, and the parameters are set reasonably by combining relevant information. During excavation, we monitor and record the shield operation and changes in excavation parameters and mud inlet and outlet conditions and then analyze and provide feedback in time to adjust the excavation parameters. The following is an example of the construction process from 101 to 200 rings through the shantytown sensitive area to analyze the regulation and control of tunneling parameters during the construction process.

In this project, the notch pressure is taken on the basis of the theoretical calculated value plus the corrected value of 0.02 MPa when the test section is dug, and Figure 4 shows the actual notch water pressure of the shield through the shantytown. The fluctuation of the water pressure at the incision should be controlled at −10 to 10 k Pa to ensure the stability of the soil [10]. During the tunneling process, it was found that the mud and water pressure at the shield incision of the east line was greater than that of the west line, and the shield incision produced a larger uplift on the ground side, and the ground uplift in turn offset some of the strati graphic losses during the construction process.

Shield initiation and advancement speed should be controlled within a reasonable range to ensure the normal excavation of the shield. Under normal conditions, tunneling speed of shield tunneling is 15–30 mm/min [4]; the tunneling speed of shield machine in special strata should be controlled by 10–20 mm/min. The speed of crossing the shantytown section should be controlled appropriately, but not too fast, which affects the follow-up speed of synchronous grouting and easily causes the cavity behind the pipe sheet wall and causes later settlement, so the matching of tunneling speed is essential for crossing the shantytown. Therefore, matching speed of tunneling is crucial for crossing the shantytown.

Referring to the settlement control experience of Nanjing Crossing Subway Line 10 project through the powder sand layer, the speed of the shield under penetration section is controlled at 0.8∼0.9 r/min, and the speed can be increased appropriately but not more than 1.0 r/min when the propulsion speed increases and the cone entry degree exceeds 50.  Figure 5 shows the tunneling speed of the shield under the soil structure.

The tunneling process of this construction has appropriately increased the tunneling speed on the basis of ensuring uniformity and stability. By appropriately increasing the tunneling speed, the construction disturbance and stratigraphic loss can be reduced to a certain extent, thus reducing the ground settlement caused by the extrusion of the shield machine's subsequent trailer on the subterranean layer.

Cutter torque is controlled at 6–9 MN-m when crossing the shantytown, and the larger the cone penetration in the same geology, the higher the torque. When the torque gradually increases significantly when the parameters such as taper entry and speed remain unchanged, it is necessary to consider whether the tool is seriously worn, and the tool wear directly causes the torque to increase significantly, so it is necessary to stop and check the tool.  Figure 6 shows the torque diagram of the shield under the shantytown construction tool.

In the soft soil layer, the rotating speed of the cutter should not be too large; otherwise, it will cause the tool to wear out faster, and the high rotating speed will easily cause greater disturbance to the soft soil layer, and the rotating speed of the shield through the shantytown section is 0.8∼1.2 r/min, and the rotating speed can be increased appropriately when the advancing speed increases and the cone entry degree exceeds 50, but not more than 1.2 r/min. It is found that the size of the excavated clouds is reduced, thus effectively avoiding the phenomenon that the shield machine is prone to clogging the tunneling mud pipe in clay strata.

## 6. Synchronized Grouting Control

Table 2 shows the grouting rate and performance parameters per cubic meter in the excavation of the shanty section by the shield

The grouting pressure should ensure that the circumferential voids are filled and the structure of the cuttings is not damaged and deformed [11]. According to experience, the calculation of the grouting pressure can be calculated by slightly more than 0.05 MPa of the cutting pressure, and the specific setting is 0.3∼0.5 MPa [32].

The gap formed by the excavation of the shield machine and the outer diameter of the pipe is 17.41 m^3^/ring, and the filling factor of the shield through the shantytown section is 130%∼180% according to experience of similar projects. At the same time, considering the shallow overburden and the influence of shielding uplift, the amount of grouting at the top and bottom of the shield should be controlled by 2 : 1. When the curve section is dug, a comparison of the grouting volume inside and outside of the curve section shows that the outside should be slightly larger than the inside.

## 7. Post-Crossing Settlement Monitoring and Pressure Fill Grouting

The shield machine continues to carry out monitoring and measurement work within a certain period of time after crossing, and Figures 7 and 8 show the monitoring curves of surface settlement and building settlement during shield crossing, respectively.

Analysis of Figures 7 and 8 shows that the shield tunnel shows a settlement trend before the palm face approaches the incision, and due to the high grouting pressure and easy disturbance of the fine sand stratum, there is a rapid uplift of the stratum in each monitoring section during the shield tunneling process, and then the soil starts to creep, consolidate, and shrink at the same time as the shield tail grouting, and the surface settlement value decreases.

The surface settlement and building settlement during the shield crossing should be controlled within the design range. At the same time, after fully considering the requirements for environmental protection and tunnel stability, if the radar grouting behind the wall detects or finds that the ground settlement still has a large trend of change or the local strata are soft, grouting should be replenished in time. Also, the stripping state caused by shield thrust should be filled in time to improve the water stopping effect.

## 8. Conclusions

In this study, the settlement control technology is studied and control measures are proposed for the construction of mega-diameter mud and water shield through shantytowns, using Wuhan Metro Line 8 Huangpu Road Station- Xujiapang Road Station interval shield through old shantytowns as the engineering background. The conclusions are as follows.

Before the shield starts, safety assessment of existing buildings (structures) should be carried out and safety control measures should be formulated; meanwhile, the tunneling parameters should be optimized through the tunneling test section.

In the process of shield tunneling, reasonable setting of each parameter should be combined with the geological condition and surrounding environment. The fluctuation value of notch pressure should be controlled by −10∼10 kPa to ensure the stability of soil body, and the starting digging speed should not be too fast and should be controlled at 10∼20 mm/min in special sections.

The maximum uplift of the foundation of the old structure in the upper shantytown during the excavation of the oversized shield is 18 mm, and the overall settlement of the structure is controlled within 18 mm.

## Figures and Tables

**Figure 1:** Shield crossing geological section.

**Figure 2:** Tunnel and shantytown flat location map.

**Figure 3:** Relationship between surface settlement and pressure difference between soil and interior.

**Figure 4:** Actual notch water pressure.

**Figure 5:** Scavenging speed of construction of 101～200 rings under shield.

**Figure 6:** Shield torque diagram.

**Figure 7:** DC03 point longitudinal settlement cumulative duration curve.

**Figure 8:** Building cumulative settlement distribution.

**Table 1:** Shield tunneling-related technical indicators.

Shield index	Numerical value
Maximum thrust	278400 KN
Normal thrust	180038 KN
Maximum propulsion speed	50 mm/min
Rated torque of cutter head	36585 kN m
Maximum torque of cutterhead	43902 kN m
Cutter head release torque	54878 kN m

**Table 2:** Synchronous grouting ratio and performance parameters.

P. O42.5 cement (kg)	Grade II fly ash (kg)	Bentonite (kg)	Fine sand (kg)	Water-reducing agent (kg)	Drinking water (kg)	Setting time (h)	Decantation rate (%)	Stone rate (%)	Consistency (cm)	Final setting strength (MPa)
200	200	80	1250	5.3	470	6	3	97	11	3.9

## Data Availability

The dataset used in this study is available from the corresponding author upon request.
